The article "A Systematic Study on the Extraction and Image Reproduction of Ceramic Sculpture Artworks" was retracted in 2023. Reasons: signs of a paper mill; suspected computer-generated content; unreliable results or conclusions; concerns about the data.

# A Systematic Study on the Extraction and Image Reproduction of Ceramic Sculpture Artworks

**DOI:** 10.1155/2022/6752589

**Published:** 2022-08-27

**Authors:** Yuhong Wang

**Affiliations:** Anhui University of Architecture, Hefei, Anhui 230601, China

## Abstract

In order to solve the research on the extraction of ceramic sculpture artwork patterns, and, in the process of image reproduction, the problem of too few feature points in the object image, the author proposes an image stitching algorithm that combines SIFT and MSER algorithms. After comprehensively analyzing the principles, advantages, and disadvantages of the current main image stitching methods, in terms of feature matching, based on the K-D tree search algorithm, the improved BBF algorithm is used to improve the search efficiency of feature points. In order to remove the possible cracks in the stitching process, an improved multiband fusion algorithm is used to seamlessly stitch the registered images. The results show that the feature points detected by the one-dimensional normal distribution algorithm are on average 0.1%, 0.5%, 1.7%, 4.4%, and 9.2%. The algorithm combining SIFT and MSER to extract feature points can reach 3.6%, 4.6%, 8.4%, 15%, and 19.1%. The experimental results show that the algorithm proposed by the author can extract more image feature points to facilitate later image registration. The image blur phenomenon in the original image fusion algorithm is solved, and a complete and clear two-dimensional plane pattern is finally obtained.

## 1. Introduction

The concept and creative inspiration of ceramic sculpture, as a way of expression of design and creation ideas in things, are based on the feeling of real life, reflecting the current artistic value. Any kind of culture has a strong nature of the times, conforming to the development of the times and personality elements interwoven. According to the characteristics of the times and humanistic demands, ceramic sculptors achieve a ceramic sculpture in line with the cultural connotation of the times. In the modern society full of diversified factors, the creators need to cultivate excellent aesthetic quality, adhere to the mentality of pursuing perfection, and combine the national spirit and the feelings of real life in the creation. Ceramic sculpture itself is a kind of artwork with historical and cultural nature, because of its decorative and artistic value, so it is recognized by the world. The transformation of various artistic concepts has made the creation of ceramic sculptures enter a period of diversification; however, in the process of preservation of ceramic sculpture artworks, pattern extraction and reproduction are time-consuming and laborious work, and the reproduction and drawing of patterns still need to be done manually by designers.

The article "A Systematic Study on the Extraction and Image Reproduction of Ceramic Sculpture Artworks" was retracted in 2023. Reasons: signs of a paper mill; suspected computer-generated content; unreliable results or conclusions; concerns about the data.

With the development of high technology, the digitization of artworks and cultural relics is no longer a problem. With the rapid development of 3D technology, its application scope has become more and more lifelike, from cultural relic restoration, simulation manufacturing, and digital sculpture to the production of ceramic sculpture artworks. However, in the process of replicating these three-dimensional cultural relics or artworks, the 3D printing technology still pays more attention to the modeling of objects; colors and patterns are ultimately drawn by hand [1]. However, in addition to the shape, the pattern is also an important part of the artwork. The traditional pattern of ceramic sculpture has a long history and brilliant achievements, and its digital protection should be promoted, so that the culture of traditional artworks can be passed on perfectly, as shown in Figure 1.

## 2. Literature Review

Han et al., first proposed a multiband fusion method in the research. It is assumed that there are two images; in the specific fusion process, the Gaussian pyramid corresponding to the image is constructed, and then the Laplacian pyramid is built according to the relevant characteristics of the graph. The weighted average fusion is performed in each bandpass layer, and the fused image is obtained by continuously accumulating pyramids [2]. Xiang et al. invented a Harris detection operator theory, the core idea of which is based on the signal autocorrelation function; by extracting features such as small-angle rotations within image elements, a sub-pixel level of accuracy is finally achieved. The advantages of this method are reflected in the processing of image edge noise and the improvement of detection efficiency; therefore, its robustness is excellent [3]. Harahap et al. proposed the SIFT algorithm, a descriptive algorithm based on local point features in the scale space, and summarized and refined it. The essence of the SIFT algorithm is to find key points in different scale spaces and calculate the orientation of the key points. Due to the use of the Gaussian scale space and the main direction, the algorithm will not change due to the zoom, illumination, translation, and other factors of the target in the image matching, and the matching force is strong [4]. Luo et al. found that the SUSAN algorithm, the Harris algorithm, and the phase consistency algorithm have the same characteristics; that is, they can keenly perceive the scale change and affine transformation of the image, and it is difficult to extract the feature points of complex images [5]. Sabale and Bahirgonde found that although the SURF operator has many advantages in feature detection, the matching performance is close to the SIFT algorithm, and the calculation time is faster, but due to its relatively small number of features detected, it reduces the accuracy of image registration. The accuracy of image registration is reduced [6]. Jia et al. proposed detection operators for affine invariant regions, typically Harris-Affine, Hessian-Affine, most stable extremum region (MSER), etc. The performance of these detection operators against different aspects such as viewing angle, illumination, scale transformation, and rotation is compared, and it is concluded that MSER performs best in most cases [7].

The article "A Systematic Study on the Extraction and Image Reproduction of Ceramic Sculpture Artworks" was retracted in 2023. Reasons: signs of a paper mill; suspected computer-generated content; unreliable results or conclusions; concerns about the data.

Based on this background, this paper focuses on the three-dimensional pattern of ceramic sculpture artwork body, positioning for high-quality reproduction and design recreation. In-depth research on the collection and image stitching technology of the three-dimensional pattern of the ceramic body is carried out, and an image reproduction system is constructed. It realizes the whole process of digitization from shooting.

## 3. The Basic Theory of the Collection of Ceramic Sculpture Patterns and Image Stitching

In the process of image acquisition, the ceramics are evenly rotated according to the angle, the camera is fixed, and the shooting method is used to reduce the color change factor and improve the efficiency of post-image processing. The color difference of the collected images is small, and the histogram matching is used to correct the color of the image. In addition, effective and accurate image denoising, image correction, etc. must be performed on the original image to ensure pixel-level calibration accuracy between images.

When the curved ceramic is rotated, the movement of the image on the ceramic body relative to the camera is nonlinear, which makes the commonly used stitching methods not directly applicable [8].

### 3.1. Collection of Ceramic Sculpture Patterns

Generally speaking, in addition to image fusion and acquisition, image stitching technology also includes image registration and preprocessing. In order to meet different needs, a variety of processing methods can be adopted, but on a general level, the steps are almost the same, and there is no very obvious difference.  Figure 2 is the corresponding flow chart. Image acquisition is to capture real-time raw images and lay a solid foundation for panoramic stitching [9]. In general, image projection is included in addition to image correction and denoising. Image registration is to find a suitable spatial transformation and align the coordinate points at the overlap. After the images are registered, the image stitching operation can be performed. Because of grayscale differences, seams and brightness differences are prone to occur. From this perspective, after image stitching is completed, image fusion should be achieved as much as possible.

The article "A Systematic Study on the Extraction and Image Reproduction of Ceramic Sculpture Artworks" was retracted in 2023. Reasons: signs of a paper mill; suspected computer-generated content; unreliable results or conclusions; concerns about the data.

### 3.2. Extraction of Ceramic Sculpture Pattern Configuration Rules

#### 3.2.1. Pattern Contour Matching

In a few cases, when there is repeated distribution of patterns, in order to extract the hierarchical relationship of patterns, this paper uses shape upper and lower grammar to describe and match the patterns, separate the patterns, complete automatic extraction, and establish the pattern library. The shape context has the characteristics of translation, scale, and rotation invariance, which can effectively match the shape. Firstly, the histogram is used to describe the point distribution on the shape contour in polar coordinates, then the Canny operator is used to obtain the shape contour of the pattern, and a set of contour sampling points is obtained by sampling [10]. Let any grain appearance shape in the pattern be A. Any point *P*_*i*_(*x*_*i*_*y*_*i*_) on the contour of the target pattern is the origin of the reference coordinate; a logarithmic polar coordinate system is established; the ordinate logr and *θ* abscissa angle are divided into *Z* and *T*, respectively; and the entire space area is divided into *Z* × *T*. Record the number of points in the relative position of the vector from point *p*_*i*_ to other points, and its statistical distribution histogram *h*_*i*_(*k*) is called the shape context of point *p*_*i*_. The algorithm is shown in the following formula:

(1) $$\begin{array}{c} h_{i}\left(k\right)=\#\left\{p\neq :p\in \text{bin}\left(k\right)\right\}. \end{array}$$

Among them, *k*={1,2,…, *K*}, *K*=*Z* × *T*. Let any point on the contour of the pattern shape B to be matched be *q*_*j*_, calculate the matching cost *C*_*ij*_ between the histograms of the *p*_*i*_ point and the *q*_*j*_ point distribution, which is shown in the following formula:

(2) $$\begin{array}{c} C_{ij}=C\left(p_{i},q_{j}\right)=\frac{1}{2}\sum_{k-1}^{k}\frac{h_{i}\left(k\right)}{h_{j}\left(k\right)}. \end{array}$$

Among them, *h*_*i*_(*k*) and *h*_*j*_(*k*) are the values in the shape histogram of the point *p*_*i*_ on the contour of the target pattern and the point *q*_*j*_ on the contour of the pattern to be matched, respectively. In the *K*th bin, the smaller the *C*_*ij*_, the smaller the matching cost of the two points and the greater the similarity.

#### 3.2.2. Configuration Rule Extraction

According to the shape context matching method, the pattern that is most similar to the target pattern in the pattern is extracted; then, the topological structure rule is used to extract the configuration of the pattern; taking the center coordinate of the pattern as the origin, determine the coordinates of the center of each pattern in the pattern. The central coordinates of each pattern in the pattern are abstracted into points, and the paths between each point are abstracted into lines; the topology formed by these points and lines is called the pattern configuration rule. According to the pattern configuration extraction rules, the configuration rules of each pattern in the case library are extracted, and the configuration rule library is established [11].

The article "A Systematic Study on the Extraction and Image Reproduction of Ceramic Sculpture Artworks" was retracted in 2023. Reasons: signs of a paper mill; suspected computer-generated content; unreliable results or conclusions; concerns about the data.

Pattern *W*={*W*1, *W*2,…, *W*_*e*_}, where *e* is the total number of different patterns in a pair of batik patterns; pattern *W*={*W*_*e*_1, *W*_*e*_2,…, *W*_*e*_*f*} in a batik pattern, where *f* is the number of times a pattern appears in a batik pattern. According to the configuration rules extracted above, according to the number of times each pattern appears in the pattern, the positions of the patterns are marked from left to right.

### 3.3. Research on Surface Image Stitching Algorithm

#### 3.3.1. Two-Dimensional Transformation of Acquired Images

The traditional image stitching and fusion methods are based on the plane assumption, so the feature points of the image are all in the same plane. At this time, the position offset relationship can be calculated by plane geometry, but the author's research object is curved. After turning the object, the movement of the image on the object relative to the camera is nonlinear; that is, simple methods such as projection transformation cannot be used to calculate the transformed parameters after rotation, and the existing traditional methods are difficult to use. The author proposes a new method to achieve 2D transformation of acquired 3D solid images.

If the RGB image is converted into an HSI image, the luminance component and the chrominance component are separated, and many measures that can be applied to deal with the gray scale of the image can be performed in the HSI image [12]. Here is a common way of processing images in true color. As can be seen in Figure 3, the three channels of H, S, and I are used to replace the three channels of R, G, and B (the luminance component is separated from the chrominance component). Then, the gray scale of the I component is increased by the method of enhancing the grayscale image. After the above processing, the data is transferred to the R, G, and B channels and finally displayed on the display screen. The enhanced image brightness component has been enhanced, so it will be brighter than the original, with no change in hue and saturation.

The article "A Systematic Study on the Extraction and Image Reproduction of Ceramic Sculpture Artworks" was retracted in 2023. Reasons: signs of a paper mill; suspected computer-generated content; unreliable results or conclusions; concerns about the data.

In the extraction of key areas, in order to remove the influence of nonlinear transformation caused by the surface as much as possible, it is necessary to select the part of the image with relatively small curvature of the actual shooting object as much as possible and perform the splicing and fusion calculation, in order to eliminate the calculation influence caused by curvature as much as possible, but the area is too small, which will affect the selection and number of feature points. Therefore, it is very important to choose a suitable region for calculation [13]. According to the empirical data obtained from the actual test, we choose the horizontal area that accounts for three-fifths of the object for splicing and fusion calculation, and there is no requirement in the vertical direction, which also reduces the problem that the background image covers the foreground texture image during fusion. Before establishing the image transformation relationship, the author first scales the image and adjusts it to a uniform size; then, the centrally extracted image occupies three-fifths of the horizontal part of the object, which is used to extract the texture image.

The image registration algorithm based on gray value is an algorithm that compares the similarity according to the gray value of pixel points between images. This algorithm process is more complicated, and the amount of calculation is large. When performing calculations, it is necessary to perform detailed comparisons for each frame of pixels, so that accurate registration of images can be achieved. The registration algorithm based on feature points can avoid the interference of noise, and the registration speed is fast. In addition, in the process of image illumination and radiation transformation, the robustness of the algorithm can also be greatly enhanced. Among the registration algorithms based on feature points, the most representative algorithms mainly include SUSAN algorithm, Harris algorithm, phase consistency algorithm, SIFT algorithm, and SURF algorithm [14].

#### 3.3.2. MSER Feature Point Extraction

The most stable extremum region is a local affine invariant feature detector proposed by Hamad Khaleefah et al. a given series of thresholds, MSER can obtain a set of thresholded binary images; then, the adjacent threshold image and the connected area between the images are analyzed, and the MSER area is finally calculated. There are two main types of MSER regions obtained. Because the extraction process is special, MSER shows some adaptability in the process of scale change, but when the scale change is too large, the effect is not as expected. Therefore, in order to effectively reduce the influence of scale variation between images, the MSER algorithm is used to detect the scale space of images [15]. MSER is an affine invariant feature region with a lack of regularity in shape and size, for the purpose of describing it through SIFT feature descriptors in the following matching. The ellipse metric area of MSER must be calculated by area affine invariant ellipse fitting and finally converted into a unit circle by normalization.

The article "A Systematic Study on the Extraction and Image Reproduction of Ceramic Sculpture Artworks" was retracted in 2023. Reasons: signs of a paper mill; suspected computer-generated content; unreliable results or conclusions; concerns about the data.

## 4. Image Registration

After the SIFT and MSER feature vectors are generated, the next step is to perform feature matching on the SIFT feature and the MSER feature. The author uses the improved K-D (K-Dimensional) tree BBF (best bin first) algorithm to roughly match the feature points, uses RANSAC to achieve accurate matching, and calculates the transformation model. Image registration often uses the Euclidean distance of the key point feature vector, which acts as the similarity between the image and the key points of the image, and then specifies the metric. In other words, it is to arbitrarily select a feature point in the reference image, and then find the quasi-image to be matched with it, for the two feature points with the shortest Euclidean distance. If the distance quotient of the feature points is not higher than a certain threshold, the two matching points can be recognized. Assuming that the feature descriptor is N-dimensional, then the Euclidean distance between the feature descriptors *d*_*i*_ and *d*_*j*_ of the above feature points is shown in the following formula:

(3) $$\begin{array}{c} d\left(i,j\right)=\sqrt{\sum_{m=1}^{n}\left(d_{i}\left(m\right)-d_{j}\left(m\right)\right)}\text{.} \end{array}$$

### 4.1. K-D Tree Algorithm

The K-D tree algorithm is an extension of the binary search tree, which mainly includes two parts. The first refers to a recursive process, where each node represents a spatial range, which can divide data [16]. Repeatedly selecting dimensions and dividing thresholds where the nodes exist, you can obtain the corresponding child nodes and then continue to expand the results until all data points are included in the process.

### 4.2. Improvement of BBF Search Algorithm

The K-D tree nearest neighbor search algorithm takes a long time and is slow in the search of high-level data. In terms of search method, the author adopts the improved BBF search method to replace the K-D tree search method. The BBF search algorithm realizes the upgrade and transformation of the K-D tree search algorithm to a large extent. It is based on the K-D tree. The priority level is used to clarify the distance of the queried node, the content is searched in an increasing order, and the closest distance is specified [17, 18]. When checking the content of some nodes, the K-D tree search algorithm takes a lot of time, and only some nodes meet the relevant requirements in the final result. In order to improve the accuracy of the results, the nearest neighbor algorithm can be used; thus, the number of nodes is limited to reduce the search time. To be in a K-D tree, search and match the nearest and next nearest eigenvalues. To get the best results, start at the root node and search to the left to identify the least-precedence sequence. Otherwise, the search starts from the right side, and finally the child node is searched. Select the content of the minimum priority sequence queue to obtain the minimum key value, and repeat the above operation content, until the content of the queue is empty; the nearest matching point and the second nearest matching point are obtained. In the process of searching, the BBF method adopts a traversal method, which will take a lot of time. In order to save time and improve work efficiency, related research methods have been improved, and the constraints of the minimum priority queue have been added. The feature value and node key value to be verified are matched, and the subtree is included in the minimum priority sequence when it meets the requirements, reducing the number of comparisons between the data and the minimum priority sequence in subsequent operations.

The article "A Systematic Study on the Extraction and Image Reproduction of Ceramic Sculpture Artworks" was retracted in 2023. Reasons: signs of a paper mill; suspected computer-generated content; unreliable results or conclusions; concerns about the data.

### 4.3. Algorithm Combining SIFT and MSER to Extract Feature Points

Among the patterns of the ceramic body, some of the patterns are line drafts, and the background is similar to a solid color; this part of the pattern is cut out, as shown in Figure 4. It is conducive to the reuse of ceramic patterns, and it is also convenient for copying [19, 20]. To extract texture patterns from images, it is necessary to use image matting technology; that is, in a relatively clean background, extract the required foreground texture images, and remove the useless background image; that is, put the required part of the image, an image processing algorithm separated from other parts [21].

The author's experimental study found that the research object of the surface rotation body determines that the author cannot directly use the common splicing algorithm. The author solves this problem by dividing the image foreground, extracting key regions, calculating the homography matrix and beam adjustment method, and transforming the collected image data into the same two-dimensional plane. Using the method based on image feature points to perform image registration, the specific process is as follows: Firstly, the method based on the combination of SIFT and MSER is used to extract feature points. On the basis of the K-D tree search algorithm, the improved BBF algorithm is used to roughly match the feature points, and then the RANSAC algorithm is used to eliminate mismatches. In order to achieve the goal of optimizing the data model to achieve the optimal matrix, the region to be fused is determined through coordinate transformation [22]. Finally, the author uses an improved multiband fusion algorithm to complete the image stitching [23]. In addition, in order to facilitate the design and recreation of some patterns, the author adopts a mapping algorithm based on real-time shared sampling. As shown in Figure 5, the pattern of simple background color is matted, and the effect is good [24].

The article "A Systematic Study on the Extraction and Image Reproduction of Ceramic Sculpture Artworks" was retracted in 2023. Reasons: signs of a paper mill; suspected computer-generated content; unreliable results or conclusions; concerns about the data.

The author has conducted many experiments on representative feature algorithms, such as SUSAN algorithm, Harris algorithm, SIFT algorithm, and SURF algorithm. Due to the particularity of the author's research objects, there are many blank patterns on the ceramic body, many non-feature points, and various types of ceramics. The SIFT algorithm has strong matching ability and can detect more feature points, MSER has better performance against image transformation, and SIFT and MSER are complementary in spatial position when extracting feature points, which can effectively improve the effect of image registration [25, 26].

It can be seen from the experimental result (Figure 6) that the average feature points detected by the one-dimensional normal distribution algorithm are 0.1%, 0.5%, 1.7%, 4.4%, and 9.2% and the combined algorithm of SIFT and MSER to extract feature points can reach 3.6%, 4.6%, 8.4%, 15%, and 19.1%. The results show that the algorithm proposed by the author can accurately achieve image stitching and, to a certain extent, can eliminate the uneven brightness of the image.

The specific analysis is as follows: (1) The quality of the collected images is good, and the effect of image stitching will be better. The quality of the images collected in different shooting environments is different, and the images collected in the studio are less disturbed, which is suitable for post-image stitching. The images collected outdoors are greatly disturbed, and more time is needed to perform image denoising, image enhancement, and other processing in the image preprocessing stage to improve the quality of the source image, which is beneficial to the stitching of the later images. (2) By analyzing the research object, repeating the experiment, and constantly modifying the algorithm, the author's splicing algorithm is finally proposed. The experimental results show that for the extraction and splicing of ceramic body patterns, the algorithm proposed by the author can improve the final splicing quality. However, for the improvement of stitching quality, the author is still exploring experiments. Reducing the loss of two-dimensional processing on image pixels, changing the algorithm to find more feature points to improve the matching accuracy, and finding a better fusion algorithm are the experimental directions of this paper. (3) The variety of ceramic types also greatly affects the quality of the splicing. (4) According to the experimental object and experimental purpose proposed by the author, the experimental effect proposed by the author is better. Moreover, the operation of removing the background color of the pattern is conducive to the reproduction and redesign of the pattern [27].

The article "A Systematic Study on the Extraction and Image Reproduction of Ceramic Sculpture Artworks" was retracted in 2023. Reasons: signs of a paper mill; suspected computer-generated content; unreliable results or conclusions; concerns about the data.

## 5. Conclusion

The digitization of artworks is the current research hotspot. Traditional ceramic sculpture artwork has high artistic value and is famous all over the world. More researchers focus their attention and research on the digitization of ceramic bodies, and fewer people pay attention to the digitization of ceramic body patterns. Therefore, the content studied by the author has important practical significance and practical application value for the protection, reproduction, dissemination, and promotion of ceramic sculpture artworks and body patterns.

## Figures and Tables

**Figure 1:** Extraction of ceramic sculpture artwork pattern.

**Figure 2:** The basic process of image stitching.

**Figure 3:** True color enhancement processing flow.

**Figure 4:** Cutout algorithm based on real-time shared sampling.

**Figure 5:** Stereo image 2Dization algorithm.

**Figure 6:** Schematic diagram of Gaussian function.

## Data Availability

The data used to support the findings of this study are available from the author upon request.
